The article "Effectiveness of Perioperative Comprehensive Evaluation of Hip Fracture in the Elderly" was published in 2022. Journal: Comput Intell Neurosci.

# Effectiveness of Perioperative Comprehensive Evaluation of Hip Fracture in the Elderly

**DOI:** 10.1155/2022/4124354

**Published:** 2022-08-05

**Authors:** Tao Zhu, Jun Yu, Ye Ma, Yue Qin, Nan Li, Haibo Yang

**Affiliations:** ^1^Department of Trauma Orthopedics, General Hospital of Ningxia Medical University, Ningxia, China; ^2^Ningxia Medical University, Yinchuan 750004, China

## Abstract

**Objective:**

The objective is to observe the effect of Comprehensive Geriatric Assessment (CGA) in the perioperative period of hip fracture.

**Methods:**

From October 2018 to October 2021, 155 patients over the age of 65 diagnosed with hip fracture and treated with surgery at the Department of Trauma Orthopaedics of General Hospital of Ningxia Medical University were randomly divided into two groups using a prospective research method. A total of 70 cases in the CGA group received a perioperative comprehensive assessment of the geriatric, and 85 cases in the control group received routine medical consultation.

**Results:**

Elderly patients with hip fractures have a high comorbidity index. Patients with abnormal daily activity before injury accounted for 55%, the abnormal rate of nutrition was 58.1%, the abnormal rate of cognition, anxiety, and depression was 81.8%, and 77.3% of the patients were in a weak state. There was no significant difference in age, gender, ASA grade, fracture type, and operation mode between the two groups, but there were significant differences in operation rate at 48 h (*χ*^2^ = 22.153; *P* ≤ 0.001), preoperative waiting time (*Z* = −6.387; *P* ≤ 0.001), total hospital stay (*Z* = −11.756; *P* ≤ 0.001), and incidence of postoperative delirium (*χ*^2^ = 23.897; *P* ≤ 0.001).

**Conclusions:**

The implementation of CGA shortened the preoperative waiting time and total hospital stay, increased the 48 h operation rate, and reduced the incidence of postoperative delirium.

## 1. Introduction

The number of elderly patients with osteoporotic fractures is increasing, and this type of elderly hip fracture seriously affects the quality of life and even the survival rate of patients. Early surgical treatment is advocated for elderly hip fractures. Some guidelines and consensus suggest that surgery should be performed within 48 hours, which can reduce the complications of long-term bed rest and postoperative mortality [1]. However, the difficulty in the treatment of such fractures is the comprehensive treatment and treatment in the perioperative period. Elderly hip fracture patients are often complicated with a variety of basic medical diseases. Some patients take a variety of drugs for a long time, which makes it difficult for orthopedic doctors to deal with them during the perioperative period and also becomes an important reason for delaying surgery [2]. At present, the treatment mode advocated is the multidisciplinary cooperation mode between orthopedics doctors and internal medicine and anesthesiologists and even the co-management mode between geriatrics and orthopedics, so as to learn from each other's strengths and make up for their weaknesses in treatment, effectively reducing the preoperative waiting time and total hospital stay, so as to provide the treatment efficiency of hip fractures in the elderly [3]. Comprehensive geriatric assessment (CGA) is a multidisciplinary evaluation and treatment model that can make rapid adjustments to meet the operation conditions, reduce unnecessary preoperative examinations, improve the operation rate within 48 hours, reduce the total length of hospital stay, improve the daily activity score before discharge, and lower the incidence of postoperative delirium [4]. In this study, the elderly comprehensive evaluation method was used to evaluate the perioperative period of elderly hip fracture patients, and the patients with abnormal scores or high-risk patients were mainly intervened in order to observe the effect of the application of the CGA method in the perioperative period of hip fracture.

The article "Effectiveness of Perioperative Comprehensive Evaluation of Hip Fracture in the Elderly" was published in 2022. Journal: Comput Intell Neurosci.

## 2. Materials and Methods

### 2.1. Inclusion Criteria

Inclusion criteria include the following: (1) age greater than 65 years old; (2) the diagnosis was femoral neck fracture, intertrochanteric fracture of the femur, or fracture of the lesser trochanter; (3) clinical symptoms and imaging data were diagnosed as a hip fracture; and (4) family members and patients agreed to participate in this study.

### 2.2. Exclusion Criteria

The exclusion criteria include the following: (1) pathological fracture; (2) old fracture; (3) multiple fractures; and (4) patients with contraindications or failure to complete the operation. This study was reviewed and approved by the ethics committee of the General Hospital of Ningxia Medical University. All subjects were informed of the study and signed informed consent.

### 2.3. Case Source

From October 2018 to October 2021, 155 patients over 65 years of age were diagnosed with hip fracture and received surgical treatment in the orthopedic department of the General Hospital of Ningxia Medical University. The patients were divided into two groups according to the random number table method. A total of 70 cases in the CGA group received perioperative elderly comprehensive evaluation. There were 85 cases in the control group. After the two groups met the operation conditions, the operation was arranged as soon as possible and completed within 48 hours of hospitalization. There was no significant difference between the two groups in age, gender, ASA grade, fracture type and operation mode (Table 1).

The article "Effectiveness of Perioperative Comprehensive Evaluation of Hip Fracture in the Elderly" was published in 2022. Journal: Comput Intell Neurosci.

### 2.4. Operation

After admission, routine examination is improved and surgical contraindications are improved; after CGA evaluation or medical consultation, surgery was performed. Closed reduction and cannulated screw fixation were used in patients with nondisplaced femoral neck fractures [5]. The displaced type was treated with half hip or total hip arthroplasty. Intramedullary or extramedullary fixation was used in patients with an intertrochanteric fracture [6]. The unstable type was treated with intramedullary fixation.

### 2.5. Contents of Comprehensive Evaluation and Intervention Measures for the Elderly

The geriatrician completes the geriatric comprehensive evaluation and records the evaluation form. Corresponding intervention measures should be taken for high-risk patients. The contents include the following. (1) Assessment of basic medical diseases: comprehensively understand the basic medical diseases of patients, quickly adjust the internal medical diseases to meet the operation conditions, reduce the waiting time and times of consultation, and reduce unnecessary preoperative examination. (2) Mini-Nutritional Assessment (MNA-SF score): enteral nutrition support should be provided to patients with malnutrition (≤11), to promote rapid postoperative recovery. [7] (3) Physical activity assessment (Bathel ADL score): for patients at a high risk of postoperative falls (≤60), effective prevention or intervention shall be carried out by means of education, rehabilitation assistance, and application of fall prevention tools by orthopedic doctors and nurses. (4) Cognitive function was assessed by Mini-cog score and MMSE score, and anxiety and depression. Anesthesiologists and orthopaedics doctors should reduce the use of benzodiazepines and opioid analgesics during or after surgery for patients with high risk of delirium, poor postoperative cognitive function (Mini-cog: ≥1, MMSE: ≤17), anxiety (SAS: ≤50), and depression (SAS: ≤ 52). Early psychological consultation and drug intervention (olanzapine and droperidol) were performed, while increasing the company of family members. Try to minimize intervention by transferring to the intensive care unit. V. Frail assessment (FRAIL score): for patients with frail status (≥3), strengthen nutritional status, strengthen rehabilitation exercise [8], strengthen nursing, and prevent falling again after the operation.

### 2.6. Diagnostic Criteria of Delirium

According to the diagnostic criteria of Diagnostic and Statistical Manual of mental disorder (Fourth revision) that delirium can be diagnosed if the following criteria are met: acute onset and fluctuating condition, inattention, disordered thinking, and the level of consciousness changes. Delirium can be diagnosed by having 1 and 2 and meeting 3 and 4. Postoperative delirium can be diagnosed from the day after the operation to the 7th day after the operation [9].

The article "Effectiveness of Perioperative Comprehensive Evaluation of Hip Fracture in the Elderly" was published in 2022. Journal: Comput Intell Neurosci.

### 2.7. Postoperative Follow-Up

After the operation, the patients were followed-up by telephone or outpatient reexamination, took X-rays until the fracture healed, guided the hip functional exercise, and followed-up until the fracture healed.

### 2.8. Statistical Analysis

The Kolmogorov–Smirnov test is used to judge whether the measurement data conform to the normal distribution. The *t*-test is used for continuous measurement data and meeting normal distribution. The Mann–Whitney U rank sum test was used for comparison between measurement data groups that did not conform to normal distribution. Pearson is used for classified data *χ*^2^ inspection. The data were statistically analyzed by SPSS20.0 analysis software. *P* < 0.05 was statistically significant.

## 3. Results

### 3.1. Comorbid State

There was no significant difference between the CGA group and the control group. However, the results showed that the patients had a high comorbidity index (Table 2).

### 3.2. CGA of Hip Fracture

Part of the evaluation content is due to the patient's dementia or inability to understand and cooperate to complete the evaluation scale. The patients had abnormal daily activity before the injury was 55%, the abnormal rate of nutrition was 58.1%, the abnormal rate of psychological assessment such as cognition, anxiety, and depression was 81.8%, and the patients in a weak state were 77.3% (Table 3).

### 3.3. 48 h Operation Rate, Preoperative Waiting, Length of Hospital Stay, Incidence of Postoperative Delirium, and ADL Score before Discharge

There were significant differences between the two groups in 48 h operation rate, preoperative waiting time, total hospital stay, and incidence of postoperative delirium (Table 4).

The implementation of geriatric comprehensive evaluation can improve the orthopadic doctors' judgment of the overall situation of patients, quantitatively evaluate the basic diseases, comorbid states, activity ability, nutrition, cognitive anxiety, depression, and weakness, and implement targeted preventive intervention and treatment measures, so as to finally improve the 48 h operation rate and shorten the preoperative waiting and total hospitalization time and can reduce the incidence of postoperative delirium. However, there was no significant difference in ADL scores between the two groups before discharge (Table 4).

The article "Effectiveness of Perioperative Comprehensive Evaluation of Hip Fracture in the Elderly" was published in 2022. Journal: Comput Intell Neurosci.

## 4. Discussion

The incidence of hip fracture in the elderly is gradually increasing [10], with a long hospital stay, high medical cost, high incidence of complications, and high mortality, which brings a serious economic and human burden to the family and the country. According to the AAOS guidelines in the United States and the consensus of experts in the diagnosis and treatment of elderly hip fractures in China [11, 12], the operation of fractures within 48 hours can reduce the incidence of complications and mortality. Because patients are often complicated with a variety of internal diseases, they need internal consultation and stabilization of internal diseases. Before the operation, they need a variety of examinations and reconsultations. In addition, oral anticoagulants are an important reason for the delay in operation [13, 14]. In order to reduce the waiting time before an operation, Grigoryan et al. [15] analyzed and summarized 18 studies and found that the cooperative treatment of elderly hip fractures by orthopedics and geriatric doctors can shorten the length of hospital stay and reduce in-hospital mortality and long-term mortality. Wu et al. [16] and others proposed that the joint management mode of orthopedics and geriatrics can shorten the preoperative waiting time and hospitalization time of patients and improve the treatment efficiency of hip fractures in the elderly. In addition, studies by Wu and others have shown that the application of the multidisciplinary cooperation model can shorten the preoperative stay in bed days, total hospital stay, postoperative out of bed activity time of elderly hip fracture patients, reduce hospitalization expenses and postoperative complications, and is more conducive to the recovery of hip function than the traditional model. In order to be more standardized and normalized, our research method was adjusted with reference to the 2018 China Guideline for the Diagnosis and Treatment of Senile Osteoporosis. During the research process, standardize the process according to the requirements of the guide at any time [17]. The above studies show that geriatrics or multidisciplinary cooperation can improve the treatment efficiency of hip fractures in the elderly and shorten the length of hospital stay and reduce the mortality rate [18]. Through routine preoperative CGA, this study can more comprehensively grasp the general situation of patients, reduce the number of consultations and waiting time, and reduce unnecessary preoperative examinations, so as to improve the 48 h operation rate and shorten the preoperative waiting time and total hospitalization time. Through the data, it can be found that the implementation of CGA can improve the 48 h operation rate to 28.6%, but the proportion is still not high. The reasons may be the lack of establishment of an emergency hospitalization or operation green channel [19], delayed evaluation, delayed operation on weekends, and other factors. The total length of stay was shortened to 20.8 days. However, compared with foreign or domestic large medical centers, it is still longer [20]. The length of stay is affected by many factors, including not only medical factors but also certain social factors [21].

The article "Effectiveness of Perioperative Comprehensive Evaluation of Hip Fracture in the Elderly" was published in 2022. Journal: Comput Intell Neurosci.

Delirium is a common complication after hip fracture surgery in the elderly [22]. It can not only prolong the hospital stay and increase medical expenses but also induce dementia and seriously affect the rehabilitation of patients [23]. The pathogenesis of delirium is unclear, but preoperative targeted prevention and intervention is an effective prevention and treatment measure. CGA is a multidisciplinary evaluation and treatment model. Through the comprehensive evaluation of elderly patients, we comprehensively collect the physical, mental, and other information needs of elderly patients, including medical evaluation (disease diagnosis, elderly complications, and multiple drugs), physical ability evaluation (self-care ability, mobility, and balance ability), and psychopsychological evaluation, socioeconomic factors, and environmental evaluation. CGA is not only for the disease itself but also for the overall situation of elderly patients [24] and not only pays attention to physical conditions but also pays more attention to cognitive and psychological conditions [25, 26]. At present, the perioperative intervention effect of CGA on elderly hip fracture patients is not consistent, and there are very few studies on CGA in China [27]. For hip fracture patients over 65 years old, the implementation of CGA can reduce the mortality rate compared with the conventional group. Forni et al. [28] performed CGA on hip fracture patients over 70 years old with surgical treatment, which can reduce the mortality rate, shorten the length of hospital stay, and reduce the rate of functional loss. Hempenius et al. [28, 29] showed that the implementation of CGA for elderly hip fractures can reduce the incidence of postoperative delirium. The above results fully show that CGA can reduce the incidence of delirium after hip fracture in the elderly, reduce postoperative mortality, and reduce the loss of hip function. This study also found that CGA can evaluate the high-risk group of postoperative delirium before the operation, and effective treatment measures and targeted drugs can reduce the incidence of postoperative delirium.

The article "Effectiveness of Perioperative Comprehensive Evaluation of Hip Fracture in the Elderly" was published in 2022. Journal: Comput Intell Neurosci.

## 5. Conclusions

CGA is an important adjuvant therapy tool in geriatrics. The results of this study show the advantages of CGA in the application of elderly hip fracture patients so that orthopedics doctors can more comprehensively grasp the overall situation of the elderly, evaluate and adjust to meet the operating conditions in the shortest time, reduce unnecessary consultation time, wait, and unnecessary preoperative examination, and improve the treatment efficiency of elderly hip fracture, which is worthy of clinical promotion.

## Figures and Tables

**Table 1:** Comparison of general data between the study group and the control group.

Project	CGA group	Study group	*χ * ^2^ * /Z*	*P*
Cases	70	85	—	—
Gender (female, %)	70.8	70.8	*χ * ^2^ = 0.227	0.634^a^
Age (years)	79.5	81.8	*Z* = −0.658	0.511^b^
ASA (I, II/III, IV)	42/28 (60/40)	56/29 (65.9/34.1)	*χ * ^2^ = 0.233	0.629^a^
Femoral neck/intertrochanteric fracture (cases, %)	37/33 (52.9/47.1)	40/45 (47.1/52.9)	*χ * ^2^ = 0.233	0.629^a^
Operation mode				
Femoral neck fracture				
Cannulated screw (cases, %)	2 (5.4)	3 (7.5)	*χ * ^2^ = 2.542	0.111^a^
Hemiarthroplasty (cases, %)	29 (78.4)	29 (72.5)		
Total hip replacement (cases, %)	6 (16.2)	8 (20.0)		
Intertrochanteric fracture				
DHS (cases, %)	3 (9.0)	1 (2.2)	*χ * ^2^ = 2.542	0.111
Intramedullary nail (cases, %)	30 (91.0)	44 (97.8)		

*Note*. a: *χ*^2^ inspection; b: Mann–Whitney *U* test.

**Table 2:** Comparison of patients in study group and control group with diseases in internal medicine (cases, %).

Complicated with medical diseases	CGA group	Study group	*χ * ^2^	*P* value
Cardiovascular diseases	37 (52.9)	40 (47.1)	0.011	0.917
Respiratory diseases	11 (15.7)	15 (17.6)	0.471	0.492
Endocrine system diseases	21 (30.0)	19 (22.4)	0.341	0.559
Neurological and psychiatric diseases	30 (42.9)	28 (32.9)	0.376	0.540
Diseases of urinary system	8 (11.4)	6 (7.1)	0.459	0.498
Digestive system diseases	7 (10.0)	4 (4.7)	0.700	0.403
Combined with a medical disease	13 (18.6)	14 (16.5)	0.001	0.969
2 kinds	20 (25.0)	22 (25.9)	0.017	0.897
3 kinds	13 (28.6)	13 (15.3)	0.028	0.866
4 or more	7 (10.0)	6 (7.1)	0.162	0.687

**Table 3:** CGA evaluation of elderly hip fracture in study group and control group.

Assessment instrument	Cases	Median score (range)	Abnormal proportion (%)
ADL	75	65.0 (0～85)	55
MNA-SF	78	6.5 (3～20)	58.1
MMSE	55	13.5 (0～29)	81.8
SAS	53	45.0 (33～66)	18.9
SDS	53	48.5 (23～79)	68.2
FRAIL	53	3.0 (0～4)	77.3

**Table 4:** Comparison of 48 h operation rate, preoperative waiting, hospital stay, incidence of postoperative delirium, and ADL score between the CGA group and the general group.

Classification	CGA group	Study group	*χ * ^2^/*Z*	*P* value
48 h operation rate (cases, %)	23 (32.9)	10 (11.8)	*χ * ^2^ = 22.153	≤0.001^a^
Preoperative waiting (d)	5.9	8.7	*Z* = −6.387	≤0.001^b^
Hospital stay (d)	20.8	23.6	*Z* = −11.756	≤0.001^b^
Incidence of postoperative delirium (%)	15 (21.4)	27 (31.8)	*χ * ^2^ = 23.897	≤0.001^a^
ADL score (score)	50.5	51.7	*Z* = −0.640	0.522^b^

*Note*. a: *χ*^2^ inspection; b: Mann–Whitney *U* test.

The article "Effectiveness of Perioperative Comprehensive Evaluation of Hip Fracture in the Elderly" was published in 2022. Journal: Comput Intell Neurosci.

## Data Availability

The datasets used and analyzed during the current study are available from the corresponding author upon reasonable request.

## References

[1] Walker J. F., Yang Y., Moore M. J. (2017). Widespread paleopolyploidy, gene tree conflict, and recalcitrant relationships among the carnivorous Caryophyllales. *American Journal of Botany*.

[2] Pajulammi H. M., Pihlajamäki H. K., Luukkaala T. H., Jousmaki J. J., Jokipii P. H., Nuotio M. S. (2017). The effect of an in-hospital comprehensive geriatric assessment on short-term mortality during orthogeriatric hip fracture program-which patients benefit the most?. *Geriatr Orthop Surg Rehabil*.

[3] Biber R., Singler K., Curschmann-Horter M., Wicklein S., Sieber C., Bail H. J. (2013). Implementation of a co-managed Geriatric Fracture Center reduces hospital stay and time-to-operation in elderly femoral neck fracture patients. *Archives of Orthopaedic and Traumatic Surgery*.

[4] Zhou Y., Rui Y., Lu P. (2020). [Research progress of multidisciplinary team co-management models for geriatric hip fracture treatment]. *Zhongguo Xiu Fu Chong Jian Wai Ke Za Zhi*.

[5] Rui Y., Qiu X., Zou J. (2019). [Clinical application of multidisciplinary team co-management in geriatric hip fractures]. *Zhongguo Xiu Fu Chong Jian Wai Ke Za Zhi*.

[6] Zhou Y., Ni Y., Li X., Chen H., Rui Y. (2019). [Research progress in treatment of femoral neck fracture in the elderly]. *Zhongguo Xiu Fu Chong Jian Wai Ke Za Zhi*.

[7] Zeng C., Lane N. E., Englund M. (2019). In-hospital mortality after hip arthroplasty in China: analysis of a large national database. *The Bone & Joint Journal*.

[8] Baroni M., Serra R., Boccardi V. (2019). The orthogeriatric comanagement improves clinical outcomes of hip fracture in older adults. *Osteoporosis International*.

[9] Hecht G., Slee C. A., Goodell P. B., Taylor S. L., Wolinsky P. R. (2019). Predictive modeling for geriatric hip fracture patients: early surgery and delirium have the largest influence on length of stay. *Journal of the American Academy of Orthopaedic Surgeons*.

[10] Jiang Y., Luo Y., Lyu H. (2021). Trends in comorbidities and postoperative complications of geriatric hip fracture patients from 2000 to 2019: results from a hip fracture cohort in a tertiary hospital. *Orthopaedic Surgery*.

The article "Effectiveness of Perioperative Comprehensive Evaluation of Hip Fracture in the Elderly" was published in 2022. Journal: Comput Intell Neurosci.

[11] Kusen J. Q., Schafroth B., Poblete B. (2019). The implementation of a Geriatric Fracture Centre for hip fractures to reduce mortality and morbidity: an observational study. *Archives of Orthopaedic and Traumatic Surgery*.

[12] Gregersen M., Mørch M. M., Hougaard K., Damsgaard E. M. (2012). Geriatric intervention in elderly patients with hip fracture in an orthopedic ward. *J Inj Violence Res*.

[13] Xing F., Chen W., Long C., Huang F., Wang G., Xiang Z. (2020). Postoperative outcomes of tranexamic acid use in geriatric trauma patients treated with proximal femoral intramedullary nails: a systematic review and meta-analysis. *Orthopaedics and Traumatology: Surgery & Research*.

[14] Christiano A. V., Elsevier H. C., Sarker S., Agriantonis G., Joseph D., Hasija R. (2021). Improving outcomes after hip fracture at a safety net hospital with a standardised hip fracture protocol. *HIP International*.

[15] Grigoryan K. V., Javedan H., Rudolph J. L. (2014). Orthogeriatric care models and outcomes in hip fracture patients: a systematic review and meta-analysis. *Journal of Orthopaedic Trauma*.

[16] Wu X., Yang M., Zhang P. (2017). Geriatric orthopedic co-management reduces time-to-operation and hospital stay in geriatric hip frac-ture patients. *J Clin Odthop Re*.

[17] Yuanzheng M., Yipeng W., Qiang L. (2018). China guideline for the diagnosis and treatment of senile osteoporosis. *Chinese Journal of Practical Internal Medicine*.

[18] Soong C., Cram P., Chezar K. (2016). Impact of an integrated hip fracture inpatient program on length of stay and costs. *Journal of Orthopaedic Trauma*.

[19] Wang C., Chang Y., Zheng Y. (2019). [Application of multidisciplinary doctor-nurse collaboration team on the perioperation management of geriatric hip fractures]. *Zhongguo Xiu Fu Chong Jian Wai Ke Za Zhi*.

[20] Van Heghe A., Mordant G., Dupont J., Dejaeger M., Laurent M. R., Gielen E. (2021). Effects of orthogeriatric care models on outcomes of hip fracture patients: a systematic review and meta-analysis. *Calcified Tissue International*.

[21] Loizzo M., Gallo F., Caruso D. (2018). Reducing complications and overall healthcare costs of hip fracture management: a retrospective study on the application of a Diagnostic Therapeutic Pathway in the Cosenza General Hospital. *Ann Ig*.

[22] Bliemel C., Oberkircher L., Eschbach D. A. (2015). Impact of Parkinson’s disease on the acute care treatment and medium-term functional outcome in geriatric hip fracture patients. *Archives of Orthopaedic and Traumatic Surgery*.

[23] Heyzer L., Ramason R., Molina J. A. D. C., Chan W. W. L., Loong C. Y., Kwek E. (2021). Integrated hip fracture care pathway (IHFCP): reducing complications and improving outcomes. *Singapore Medical Journal*.

The article "Effectiveness of Perioperative Comprehensive Evaluation of Hip Fracture in the Elderly" was published in 2022. Journal: Comput Intell Neurosci.

[24] Mittal C., Lee H. C. D., Goh K. S. (2018). ValuedCare program: a population health model for the delivery of evidence-based care across care continuum for hip fracture patients in Eastern Singapore. *Journal of Orthopaedic Surgery and Research*.

[25] Lynch G., Shaban R. Z., Massey D. (2015). Evaluating the orthogeriatric model of care at an Australian tertiary hospital. *International Journal of Orthopaedic and Trauma Nursing*.

[26] Milisen K., Foreman M. D., Abraham I. L. (2001). A nurse-led interdisciplinary intervention program for delirium in elderly hip-fracture patients. *Journal of the American Geriatrics Society*.

[27] Roberts H. J., Barry J., Nguyen K. (2021). 2021 John Charnley Award: a protocol-based strategy when using hemiarthroplasty or total hip arthroplasty for femoral neck fractures decreases mortality, length of stay, and complications. *The Bone & Joint Journal*.

[28] Forni S., Pieralli F., Sergi A., Lorini C., Bonaccorsi G., Vannucci A. (2016). Mortality after hip fracture in the elderly: the role of a multidisciplinary approach and time to surgery in a retrospective observational study on 23, 973 patients. *Archives of Gerontology and Geriatrics*.

[29] Hempenius L., Slaets J. P. J., van Asselt D., de Bock G. H., Wiggers T., van Leeuwen B. L. (2013). Outcomes of a geriatric liaison intervention to prevent the development of postoperative delirium in frail elderly cancer patients: report on a multicentre, randomized, controlled trial. *PLoS One*.

